RETRACTED

# CRISPLD1 promotes gastric cancer progression by regulating the Ca^2+^/PI3K-AKT signaling pathway

**DOI:** 10.1016/j.heliyon.2024.e27569

**Published:** 2024-03-07

**Authors:** Liqiang Hu, Jianghua Shi, Zichen Zhu, Xuemei Lu, Huibo Jiang, Hanyang Yu, Hao Liu, Wei Chen

**Affiliations:** a Graduate school of Zhejiang Chinese Medical University, Hangzhou, Zhejiang, China; b Cancer Institute of Integrated Traditional Chinese and Western Medicine, Key Laboratory of Cancer Prevention and Therapy Combining Traditional Chinese and Western Medicine of Zhejiang Province, Zhejiang Academy of Traditional Chinese Medicine, Hangzhou, Zhejiang, China; c School of Computer Science, University of Nottingham Ningbo China, Ningbo, China

**Keywords:** Gastric, Cancer, CRISPLD1, PI3K-AKT, Calcium

## Abstract

Gastric cancer (GC) is a malignant tumor with poor prognosis. Studies have shown that cysteine-rich secretory protein LCCL domain containing 1 (CRISPLD1) is associated with tumor progression. However, its role in GC is unclear. The present study aimed to determine the pathogenic mechanism of CRISPLD1 in GC. Analysis of public databases revealed high mRNA expression of *CRISPLD1* in GC, which was associated with poor prognosis. Additionally, *CRISPLD1* expression levels showed significant correlations with T stage, overall survival events, and stage. Knockdown of *CRISPLD1* reduced cell proliferation, invasion, and migration. Furthermore, *CRISPLD1* knockdown decreased intracellular calcium levels in GC cells and inhibited the phosphatidylinositol-4,5-bisphosphate 3-kinase (PI3K)-protein kinase B (AKT) signaling pathway. Treatment with an AKT activator reversed the inhibitory effect of *CRISPLD1* knockdown on GC cell migration and invasion. Our findings suggest that CRISPLD1 promotes tumor cell progression in GC by mediating intracellular calcium levels and activating the PI3K-AKT pathway, highlighting CRISPLD1 as a potential therapeutic target for GC.

## 1 Introduction

Gastric cancer (GC) is the fifth most prevalent cancer and ranks third in terms of cancer-related deaths globally [1,2]. The metastatic capability of GC cells is a major factor contributing to the poor prognosis of patients with GC. Current treatment options for GC include surgery, chemotherapy, and biological therapy; however, they often yield unsatisfactory results for both patients and physicians [3]. Despite advances in medical and endoscopic technologies, as well as significant progress in immunotherapy, the efficacy of therapies used to treat GC remains limited, resulting in a high mortality rate in many countries, including China [[4], [5], [6]]. In fact, GC cases in China account for approximately 42.6% of the global GC incidence and 45.0% of global gastric cancer deaths [7,8]. Therefore, the discovery of novel biomolecules and signaling pathways related to GC might lead to new therapeutic strategies.

RETRACTED

The *CRISPLD1* gene (encoding cysteine-rich secretory protein LCCL domain containing 1) is located in the chromosomal region 8q21.13. CRISPLD1 is a secreted protein that contains an LCCL domain that is rich in cysteine residues. CRISPLD1 was found in the secretome of choroid plexus epithelial cells, exosomes from human salivary glands, and prostatic secretions [9,10]. Abnormal expression of CRISPLD1 has been observed in various cancers, including acute myeloid leukemia (AML), renal cell carcinoma, and endometrial cancer, suggesting its potential as a biomarker in tumor diagnosis [[11], [12], [13]]. Our present study indicated that CRISPLD1 is aberrantly expressed in a wide range of cancers, and its expression is significantly associated with the clinical prognosis of GC. Single-gene enrichment analysis suggested that CRISPLD1 is mainly involved in the calcium and phosphatidylinositol-4,5-bisphosphate 3-kinase (PI3K)-protein kinase B (AKT) signaling pathways. The PI3K/Akt/mTOR signaling pathway plays a significant role in the development, prognosis, and metastasis of GC through various mechanisms, including inhibiting cell apoptosis, promoting chemoresistance, and inducing epithelial-mesenchymal transition(EMT) [14,15]. However, it remains unclear whether CRISPLD1 regulates tumor progression through the calcium and PI3K-AKT signaling pathways in GC.

Herein, we investigated the expression and prognostic significance of CRISPLD1 in patients with GC by analyzing data from publicly available databases. Functional assays revealed that knockdown of *CRISPLD1* significantly inhibited the proliferation, invasion, and migration of GC cells *in vitro*. Furthermore, we analyzed the relationship between CRISPLD1 and the calcium and PI3K-AKT signaling pathways. Mechanistically, downregulation of CRISPLD1 resulted in decreased intracellular calcium levels in GC cells, inhibited the activation of the PI3K-AKT signaling pathway, and suppressed GC tumor progression. Thus, CRISPLD1 might serve as a therapeutic target in patients with GC.

## 2 Materials and methods

### 2.1 Cell culture

The human gastric cancer cell lines MKN-47, MGC-803, BGC-823, and HGC-27, and the human gastric mucosal cell line GES-1 were purchased from Procell (Wuhan, China). We cultured the cells in Roswell Park Memorial Institute (RPMI)-1640 medium (Gibco, Grand Island, NY, USA), supplemented with 10% fetal bovine serum (Gibco). The cells were kept in a cell incubator at 37 °C and 5% CO_2_ to maintain optimal growth conditions.

RETRACTED

### 2.2 Bioinformatic analyses

We analyzed *CRISPLD1* expression in different cancers using the TIMER2.0 web tool (http://timer.cistrome.org/) and extracted relevant clinical expression data and patient survival information from The Cancer Genome Atlas (TCGA) database (https://cancergenome.nih.gov/). We also performed survival analysis related to *CRISPLD1* in patients with different stages of GC using the Kaplan-Meier Plotter web tool (http://kmplot.com/analysis/index.php?p=service&cancer=gastric). To validate the expression of *CRISPLD1* in GC, we utilized the GEPIA (Gene Expression Profiling Interactive Analysis) web tool (http://gepia.cancer-pku.cn/) and the UALCAN (University of Alabama at Birmingham cancer data analysis portal) database (https://ualcan.path.uab.edu/). Furthermore, we retrieved and evaluated the expression data of *CRISPLD1* in both non-tumor and tumor tissues of patients with GC from the GEO (Gene Expression Omnibus) database (GSE54129).

### 2.3 Cell transfection

We obtained small interfering RNAs (siRNAs) targeting *CRISPLD1* (si-CRISPLD1-1, CTTTGTATATGCCACTAATAA; si-CRISPLD1-2, GTATCCAACAGCCTCTAATAT; si-CRISPLD1-3, CGGTGGTTATGTTGATGTAAT) and a negative control siRNA (si-NC) from GenePharma (Shanghai, China), which were transfected into HGC-27 and BGC-823 cell lines in a 6-well plate. After incubating the cells for 24 h until they reached approximately 60% confluency, we mixed the siRNAs with Lipofectamine 2000 (Invitrogen, Waltham, MA, USA) and transfected the cells according to the manufacturer's protocol.

### 2.4 Quantitative real-time reverse transcription PCR (RT-qPCR)

To analyze the mRNA expression level of *CRISPLD1*, extracted total RNA was reverse transcribed into cDNA using a PrimeScript™ RT Reagent Kit (Takara, Shiga, Japan) and then conducted quantitative real-time PCR (qPCR) analysis using the cDNA as the template and a TB Green Premix Ex Taq™ kit (Takara), according to the supplier's protocol. The reaction conditions were: 95 °C for 30 s, followed by 40 cycles of 95 °C for 5 s and 60 °C for 30 s. We used the β-actin gene (*ACTB*) as an internal control and calculated the relative expression level using the 2^−ΔΔCT^ method. The primer sequences for *CRISPLD1* and *ACTB* were as follows: *CRISPLD1* (F: 5′-GTGACTTGTGAAACAACTGTG-3'; R: 5′-ACGAGGACAGTATACTCTTGG-3′) and *ACTB* (F: 5′-TGGCACCCAGCACAATGAA-3'; R: 5′-CTAAGTCATAGTCCGCCTAGAAGCA-3′), which were synthesized by GenePharma.

### 2.5 Western blotting

Proteins were extracted from cells using Radioimmunoprecipitation assay (RIPA) lysis buffer (Beyotime, Jiangsu, China) and quantified using a bicinchoninic acid (BCA) protein assay kit (Thermo Fisher Scientific, Waltham, MA, USA). The extracted proteins were then separated using sodium dodecyl sulfate-polyacrylamide gel electrophoresis (SDS-PAGE) and transferred onto polyvinylidene fluoride (PVDF) membranes (Millipore, Billerica, MA, USA), which were blocked using 5% skim milk. The PVDF membranes were then incubated with primary antibodies recognizing glyceraldehyde-3-phosphate dehydrogenase (GAPDH) (1:5000, CST, Danvers, MA, USA), AKT (1:1000, CST), phosphorylated (p)-AKT (1:1000, CST), PI3K (1:1000, CST), and p-PI3K (1:1000, CST) antibodies at 4 °C overnight. Next day, the membranes were incubated with horseradish peroxidase-conjugated secondary antibodies (Beyotime, Jiangsu, China). The immunoreactive protein bands were visualized using a chemiluminescence (ECL) detection kit (Solarbio, Beijing, China) and imaged using the ChemiDoc™ XRS imaging system (Bio-Rad, Hercules, CA,USA).

RETRACTED

### 2.6 Cell counting kit 8 (CCK-8) assay

After transfection with siRNAs, the HGC-27 and BGC-823 cells were digested with trypsin and resuspended in fresh culture medium at a concentration of 4 × 10^4^ cells/ml. The cells were subsequently seeded into a 96-well plate at a volume of 100 μl per well, with six replicates for each group, and this process was repeated three times for biological replication. The plate was incubated at 37 °C and 5% CO_2_ for 24, 48, 72, and 96 h. Thereafter, 10 μl of CCK-8 reagent (Dojindo, Kumamoto, Japan) was added to each well, and the cells were further incubated for 3 h. The absorbance of each well was measured at 450 nm using an enzyme-linked immunosorbent assay reader (Bio-Rad).

### 2.7 Colony formation assay

Following siRNA transfection, HGC-27 and BGC-823 cells were digested with trypsin and seeded into 6-well plates at a density of 1 × 10^4^ cells/ml, . The cells were cultured in fresh medium for 14 days, with medium replacement every 3 days, to allow colony formation. After the incubation period, the cells were fixed using 4% paraformaldehyde, stained with 0.5% crystal violet, and the number of colonies was counted under a microscope after washing with phosphate-buffered saline (PBS).

### 2.8 Wound-healing assay

Following siRNA transfection, HGC-27 and BGC-823 cells were seeded into 6-well plates at a concentration of 1 × 10^6^ cells/ml. After overnight incubation in serum-free medium, a scratch was created on the cell monolayer using a pipette tip, and the width of the scratch was imaged and measured. The cells were then incubated for an additional 48 h, after which the scratch was imaged and measured again to evaluate the extent of cell migration (wound healing).

### 2.9 Transwell assays

Matrigel (BD Biosciences, San Jose, CA, USA) was added to the upper chamber of a Transwell insert (Corning Inc., Corning, NY, USA) for Transwell assays. In brief, 100 μl of serum-free medium and 1 × 10^5^ cells were added to the upper chamber, while 700 μl of complete medium was added to the lower chamber. After 24 h, the cells on the underside of the membrane were fixed using 4% paraformaldehyde, stained with 0.1% crystal violet, and observed under a microscope (Nikon, Tokyo, Japan) to visualize and count the cells adhering to the lower surface.

RETRACTED

### 2.10 Immunofluorescence analysis

Cultivate cells in a 24-well plate and fix with 4% paraformaldehyde for 15 min. Wash three times and permeabilize for 10 min in PBS containing 0.2% Triton X-100. Incubate overnight at 4 °C with mouse anti-human antibodies p-AKT and p-PI3K (Proteintech, China). The next day, wash with PBS and incubate for 2 h with goat anti-mouse IgG secondary antibody labeled with Alexa Fluor 488. After washing with PBS, incubate the cell samples with DAPI for 5 min and capture fluorescence images using a fluorescence microscope.

### 2.11 Analysis of differentially expressed genes (DEGs)

To identify genes that were differentially expressed between high and low *CRISPLD1* expression groups in GC samples from the TCGA, we conducted DEG analysis using the DESeq2 package [16]. Adjusted p-values (P adj) were employed to minimize the occurrence of false positives. In this study, DEGs were selected based on the criteria of (|log2(fold-change (FC)| > 1.5, P adj <0.05). The identification of DEGs provides valuable insights into the potential roles of CRISPLD1 in GC development and progression.

### 2.12 Functional enrichment analysis

To gain insights into the potential targets and underlying mechanisms of CRISPLD1 in GC, we conducted DEG enrichment analysis using the ClusterProfiler package [17], which included gene ontology (GO) and Kyoto Encyclopedia of Genes and Genomes (KEGG) enrichment. Differentially expressed genes (DEGs) were identified by comparing the signal values between the groups, using a significance threshold of P adj <0.05 and |log2(FC)| > 1.5. Our single-gene differential analysis of *CRISPLD1* revealed that its high expression was mainly accompanied by upregulated DEGs. We selected 629 significantly upregulated DEGs for GO and KEGG analysis, which allowed us to identify enriched biological processes, molecular functions, cellular components, and the relevant signaling pathways associated with the dysregulation of *CRISPLD1* expression in GC.

### 2.13 Calcium concentration measurement

Fluo-4/acetoxymethyl (AM) fluorescence staining was used to determine the Ca^2+^ levels in HGC-27 and BGC-823 cells. Briefly, HGC-27 and BGC-823 cells transfected with siRNAs were harvested and incubated with Fluo-4/AM (1 μmol final concentration, Beyotime) at 37 °C for 40 min. The peak shift in the fluorescein isothiocyanate (FITC) channel was analyzed using a flow cytometer(BD, NJ, USA), and the level of Ca^2+^ was expressed as the mean fluorescence intensity (MFI). In addition, fluorescence microscopy (Zeiss, White Plains, NY,USA) was used to observe the cells and analyze the images to determine changes in intracellular Ca^2+^ levels.

RETRACTED

### 2.14 Statistical analysis

Statistical analysis was performed using the SPSS software (IBM Corp., Armonk, NY, USA. Comparisons between two groups were performed using two-tailed paired Student's *t*-tests and Mann-Whitney *U* test, while comparisons among multiple groups (at least three groups) were analyzed using one-way analysis of variance (ANOVA). GraphPad Prism 9.0 (GraphPad Inc., La Jolla, CA, USA) was used to prepare the statistical graphs. A P value less than 0.05 indicted statistical significance(*p < 0.05; **p < 0.01; ***p < 0.001).

## 3 Results

### 3.1 The expression level and prognostic value of *CRISPLD1* in pan-cancer

We applied the TIMER2.0 tool to analyze the expression of *CRISPLD1* in TCGA pan-cancers. Compared with that in normal tissues, the expression level of *CRISPLD1* was higher in ESCA (esophageal cancer), LUSC (lung squamous cell carcinoma), and STAD (gastric adenocarcinoma) tumor tissues (P < 0.05). The expression levels of *CRISPLD1* in BRCA (breast cancer), KICH (kidney chromophobe cells), KIRC (clear renal cell carcinoma), LIHC (hepatocellular carcinoma), SKCM (cutaneous melanoma), and THCA (thyroid cancer) were lower than those in the corresponding of control tissues (Fig. 1A). We next evaluated the impact of CRISPLD1 on patient prognosis in cancers in which it was differentially expressed. Kaplan–Meier survival plots showed that high expression of *CRISPLD1* in STAD was associated with significantly shorter overall survival (OS) (Fig. 1B). There was no significant difference in prognostic indicators in the other cancers (Fig. 1C–J). There is a large degree of heterogeneity between different cancers, with only a few tumor types, including GC, having high *CRISPLD1* expression levels, and survival analysis was significant only in GC. This suggested that CRISPLD1 is an important therapeutic target in GC.

**Fig. 1:** Expression and survival analysis associated with CRISPLD1 in different cancers. (A) Analysis of *CRISPLD1* expression in different tumors in the TCGA using the TIMER2 online database; (B–J) Kaplan-Meier survival analysis of high and low expression of *CRISPLD1* in different tumors. ***p < 0.001; **p < 0.01; *p < 0.05.

RETRACTED

### 3.2 Bioinformatic analysis of the relationship between *CRISPLD1* expression and the clinicopathological characteristics of GC

We downloaded the clinical data and gene expression data for GC in the TCGA and analyzed the relationship between *CRISPLD1* expression and clinicopathological parameters in patients with GC. The parameters analyzed include sample type (normal/tumor), T stage (T1&T2/T3&T4), M stage (M0/M1), N stage (N0&N1/N2&N3), age (≤65/> 65), pathological stage (stage I and stage II/III and IV), OS event (alive/dead). The results showed that the expression of *CRISPLD1* in GC tissues was significantly higher than that in normal samples (Fig. 2A). The expression of *CRISPLD1* in GC at the T3&T4 stage was significantly higher than that at the T1&T2 stage (Fig. 2B). In the disease OS event analysis of patients with GC, high expression of *CRISPLD1* showed an association with patient death (Fig. 2C). *CRISPLD1* was highly expressed in patients ≤65 years old (Fig. 2D). No correlation was found between *CRISPLD1* expression and M stage or N stage (Fig. 2E and F). The expression of *CRISPLD1* was significantly higher in late stage II and stage III GC samples than in early pathological stage I samples (Fig. 2G). Receiver operating characteristic (ROC) curves were drawn to determine the sensitivity and specificity of *CRISPLD1* expression in distinguishing GC tissues from the normal gastric mucosa. The results showed that the area under the ROC curve was 0.702, indicating that *CRISPLD1* expression analysis might contribute to the identification of GC tissues (Fig. 2H). The predicted role of CRISPLD1 in GC was detected using Kaplan-Meier plotter, and the results showed that high *CRISPLD1* expression in stage III and stage IV GC predicted poor patient prognosis.

**Fig. 2:** Relationship between *CRISPLD1* expression in TCGA and clinicopathological features of patients with GC and verification of CRISPLD1 expression levels in tissues and cells. (A) Analysis of *CRISPLD1* expression between normal and cancerous tissues; (B) *CRISPLD1* expression analysis between T1&T2 and T3&T4 patients with GC; (C) *CRISPLD1* expression analysis between living and deceased patients with GC; (D) Analysis of *CRISPLD1* expression among patients with GC aged 65 years or younger; (E) *CRISPLD1* expression analysis between M0 and M1 patients with GC; (F) Analysis of *CRISPLD1* expression between N0&N1 and N2&N3 patients with GC; (G) Analysis of *CRISPLD1* expression among patients with stage I, II, III, and IV GC; (H) ROC curves of *CRISPLD1* in the TCGA data; (I) The Kaplan-Meier plotter database was used to analyze CRISPLD1-related survival of patients with pathological stage I, II, III and IV GC; (J) GEPIA and (K) UALCAN databases were used to compare *CRISPLD1* mRNA expression in GC samples and normal gastric tissue samples. (L) The GEO database was utilized to assess *CRISPLD1* levels in 111 human gastric cancer tissues and 21 noncancerous gastric tissues. (M) RT-qPCR was performed to determine *CRISPLD1* mRNA levels in human gastric cancer cells and human gastric epithelial cells, means ± SD, n = 3. ***p < 0.001; **p < 0.01; *p < 0.05.

RETRACTED

### 3.3 *CRISPLD1* expression verification in tissues and cells

We applied UALCAN and GEPIA tools to analyze the expression of *CRISPLD1* in GC, and the results further confirmed that the expression of *CRISPLD1* in tumor tissues was significantly higher than that in the normal group (Fig. 2J and K). The same results were obtained using GEO data analysis (GSE54129) (Fig. 2L). The correlation analysis between clinical features of GC patients from the TCGA database and CRISPLD1 expression revealed significant associations with the T stage, race, and age of GC patients. These findings strongly suggest that CRISPLD1 has the potential to be utilized as a valuable prognostic biomarker for GC(Table 1). Therefore, we examined the expression of *CRISPLD1* in GC and normal cell lines. We performed RT-qPCR detection of *CRISPLD1* mRNA in GC cell lines and GSE-1 cells. The results showed that *CRISPLD1* mRNA levels were significantly increased in GC cell lines compared with those in GSE-1 cells(Fig. 2M). Therefore, we chose HGC-27 and BGC-823 as GC model cell lines for subsequent experiments in this study.

**Table 1:** Correlations between CRISPLD1 expression and clinicopathologic features of GC patients.

Characteristic	Low expression of CRISPLD1	High expression of CRISPLD1	p
n	187	188	
T stage, n (%)			0.033*
T1	15 (4.1%)	4 (1.1%)	
T2	43 (11.7%)	37 (10.1%)	
T3	84 (22.9%)	84 (22.9%)	
T4	43 (11.7%)	57 (15.5%)	
N stage, n (%)			0.539
N0	60 (16.8%)	51 (14.3%)	
N1	50 (14%)	47 (13.2%)	
N2	38 (10.6%)	37 (10.4%)	
N3	32 (9%)	42 (11.8%)	
M stage, n (%)			0.711
M0	165 (46.5%)	165 (46.5%)	
M1	14 (3.9%)	11 (3.1%)	
Pathologic stage, n (%)			0.050
Stage I	35 (9.9%)	18 (5.1%)	
Stage II	48 (13.6%)	63 (17.9%)	
Stage III	72 (20.5%)	78 (22.2%)	
Stage IV	20 (5.7%)	18 (5.1%)	
Race, n (%)			0.041*
Asian	42 (13%)	32 (9.9%)	
Black or African American	8 (2.5%)	3 (0.9%)	
White	105 (32.5%)	133 (41.2%)	
Age, n (%)			0.032*
≤65	71 (19.1%)	93 (25.1%)	
>65	114 (30.7%)	93 (25.1%)	

Abbreviations: T, tumor status; N, regional lymph nodes status; M, metastasis status; GC, gastric cancer.

### 3.4 CRISPLD1 regulates GC cell proliferation and migration *in vitro*

To explore the role of CRISPLD1 in GC, we used an siRNA to knock down *CRISPLD1* expression in HGC-27 and BGC-823 cell lines (Fig. 3A). A CCK-8 assay showed that knockdown of *CRISPLD1* expression significantly inhibited cell proliferation compared with that in the si-NC group (Fig. 3B). Likewise, the results of the colony formation assay showed that the number of colonies formed was significantly reduced upon knockdown of *CRISPLD1* (Fig. 3C). Next, wound healing experiments showed that knockdown of *CRISPLD1* significantly inhibited cell migration compared with the that of the si-NC group (Fig. 3D and E). Similarly, in Transwell experiments, compared with that in the si-NC group, knockdown of *CRISPLD1* significantly inhibited the cell invasion ability (Fig. 3F and G). Overall, these results indicated that higher *CRISPLD1* expression promotes GC cancer progression.

RETRACTED

**Fig. 3:** Knockdown of *CRISPLD1* inhibits the proliferation and migration of GC cells. (A) RT-qPCR detection of *CRISPLD1* expression in GC cells after si-CRISPLD1 treatment; (B) CCK8 assay to determine the viability of GC cells after *CRISPLD1* knockdown; (C) Colony formation assay to assess the clonogenic ability of GC cells after *CRISPLD1* knockdown; (D–E) Wound healing assay to evaluate the effect of *CRISPLD1* knockdown on the migration ability of GC cells; (F–G) Transwell assay demonstrating the impact of *CRISPLD1* knockdown on the invasive ability of GC cells. means ± SD, n = 3, ***p < 0.001; **p < 0.01; *p < 0.05.

### 3.5 Differential gene expression analysis and enrichment analysis

To explore the possible mechanism of CRISPLD1 in GC, DEG analysis and enrichment analysis were performed using TCGA GC samples. First, we identified DEGs between the high and low *CRISPLD1* expression GC sample groups in the TCGA data. We obtained 828 DEGs (|log2(FC)| > 1.5, P adj <0.05), including 629 upregulated genes and 199 downregulated genes. Among the DEGs, we performed GO and KEGG enrichment analysis on the 629 upregulated genes. Functional analysis of biological processes (BP) revealed that the differentially expressed genes (DEGs) are mainly enriched in the regulation of membrane potential and regulation of *trans*-synaptic signaling (Fig. 4A). Additionally, there were three notable enrichment terms in cellular components (CC), including synaptic membrane, cell-cell junction, and transmembrane transporter complex (Fig. 4B). Molecular function (MF) analysis showed that the proteins encoded by DEGs play a crucial role in enhancing the activity of signaling receptors, ion channels, metal ion transmembrane transporters, and cation channels (Fig. 4C). KEGG pathway analysis showed that the upregulated DEGs were mainly enriched in Neuroactive ligand-receptor interaction, the Calcium signaling pathway, and the PI3K-AKT signaling pathway (Fig. 4D).

RETRACTED

**Fig. 4:** GO and KEGG enrichment analysis of differentially expressed genes. (A) Bubble chart displaying the top 10 biological process (BP) terms; (B) Bubble chart presenting the top 10 cellular component (CC) terms; (C) Bubble chart illustrating the top 10 molecular function (MF) terms; (D) Bubble chart showing the significant KEGG pathway terms. means ± SD, n = 3, ***p < 0.001; **p < 0.01; *p < 0.05.

### 3.6 Knockdown of *CRISPLD1* inhibited intracellular Ca^2+^ levels and the PI3K-AKT signaling pathway in GC cells

Calcium ions are important signaling molecules in cells, which have been shown to play a critical role in regulating the malignant phenotype of tumor cells [18,19]. DEG enrichment analysis indicated that CRISPLD1 is involved in the regulation of calcium signaling in GC cells. Therefore, we investigated whether CRISPLD1 could regulate the calcium ion concentration in GC cells. We used the Fluo-4 Ca^2+^ fluorescent probe to detect the changes in Ca^2+^ levels in GC cells *in vitro*. Flow cytometry analysis showed that siRNA-mediated silencing of *CRISPLD1* reduced the concentration of Ca^2+^ in GC cells (Fig. 5A and B). Meanwhile fluorescence microscopy observation showed that knockdown of *CRISPLD1* in HGC-27 and BGC-823 cells weakened the fluorescence intensity of the Ca^2+^ fluorescent probe (Fig. 5C and D). Studies have shown that phosphatase and tensin homolog (PTEN) and cytosolic calcium homeostasis are two major upstream regulators of the AKT pathway, with multiple studies demonstrating their significant roles in regulating AKT activity [20,21]. In addition, based on KEGG analysis, we found that the PI3K-AKT signaling pathway was significantly enriched. We hypothesized that CRISPLD1 might activate activation of the PI3K-AKT signaling pathway by regulating intracellular calcium ion levels. Western blotting analysis showed that siRNA-mediated silencing of *CRISPLD1* significantly decreased the levels of p-PI3K and p-AKT in HGC-27 and BGC-823 cells, indicating that knockdown of CRISPLD1 can inhibit the activation of the PI3K-AKT signaling pathway in GC cells (Fig. 5E and F). Immunofluorescence experiments demonstrated that knockdown of *CRISPLD1* in HGC-27 and BGC-823 cells weakened the fluorescence intensity of p-AKT (Fig. 5G and H). Immunofluorescence experiments revealed that the fluorescence intensity of p-PI3K was attenuated in HGC-27 and BGC-823 cells upon knockdown of CRISPLD1(Fig. 5I and J).

**Fig. 5:** Impact of *CRISPLD1* knockdown on intracellular calcium levels and the PI3K-AKT signaling pathway. (A–B) Flow cytometry analysis of the fluorescence intensity of Fluo-4 AM in cells after *CRISPLD1* knockdown; (C–D) Fluo-4 AM calcium imaging of intracellular calcium levels after *CRISPLD1* knockdown; (E–F) Western blotting analysis of the levels of phosphorylated PI3K and AKT after *CRISPLD1* knockdown. (G–J) Immunofluorescence analysis was used to determined the expression of p-AKT and p-PI3K in HGC-27 and BGC-823 cells. means ± SD, n = 3, ***p < 0.001; **p < 0.01; *p < 0.05.

RETRACTED

### 3.7 CRISPLD1-mediated proliferation, migration, and invasion of gastric cancer cells is dependent on the PI3K-AKT signaling pathway

The role of AKT signaling in regulating tumor cell migration and invasion, including that in gastric tumors, is widely accepted [22,23]. To investigate the role of AKT in CRISPLD1-mediated proliferation, migration, and invasion of GC cells, we treated *CRISPLD1*-silenced HGC-27 and BGC-823 cells with SC79, an AKT activator. The CCK8 assay results demonstrated that SC79 treatment restored the proliferation capability of *CRISPLD1*-silenced cells (Fig. 6A). Overexpression of CRISPLD1, on the other hand, promoted gastric cancer cell proliferation, which was reversed by AKT inhibitor MK2206 (Fig. 6B). Furthermore, our scratch assay and Transwell assay results indicated that SC79 could reverse the inhibitory effects of *CRISPLD1* silencing on cell migration and invasion (Fig. 6C and E). The enhanced migration and invasion of GC cells due to CRISPLD1 overexpression were found to be counteracted by the AKT inhibitor MK2206 (Fig. 6D and F). These findings suggested that the proliferation, migration, and invasion of GC cells mediated by CRISPLD1 might be regulated by the PI3K-AKT signaling pathway.

**Fig. 6:** Reversal of the effects of CRISPLD1 on the proliferation and invasion of GC cells by SC79. (A–B) Assessment of the impact of different treatments on GC cell proliferation using the CCK8 assay; (C–D) Evaluation of cell migration ability through wound healing experiments; (E–F) Assessment of cell invasion ability through Transwell chamber assays. means ± SD, n = 3, ***p < 0.001; **p < 0.01; *p < 0.05.

### 3.8 Knockdown of CRISPLD1 inhibits growth of GC in vivo

To evaluate the impact of CRISPLD1 on in vivo proliferation of GC, stable HGC-27 cells transfected with sh-CRISPLD1 and sh-NC group were implanted into nude mice. Tumor volume was measured every 4 days after injection. During the development of xenograft tumors, the tumor volume in the sh-CRISPLD1 group was significantly smaller than the sh-NC group (Fig. 7A and B). Moreover, the average tumor weight in the sh-CRISPLD1 group was significantly lower than the sh-NC group (Fig. 7C). Additionally, histological analysis of tumor sections demonstrated that the proliferative activity of Ki-67 stained tumors was significantly reduced in the sh-CRISPLD1 group compared to the sh-NC group (Fig. 7D). These findings are consistent with our *in vitro* studies and strongly suggest that CRISPLD1 contributes to the progression of GC in vivo.

RETRACTED

**Fig. 7:** CRISPLD1 promotes tumorigenesis of gastric cancer cells in vivo. (A) Knockdown of CRISPLD1 inhibits subcutaneous tumor formation in nude mouse model. (B) Tumor volume was measured and recorded every 4 days. (C) Tumor weight was measured at the end of the experiment. (D) Immunohistochemical staining and statistical analysis of proliferation index factor Ki67 in tumor sections. means ± SD, n = 5, ***p < 0.001; **p < 0.01; *p < 0.05.

## 4 Discussion

Human GC is one of the most invasive malignant tumors and the third leading cause of cancer-related death worldwide because of its rapid progression to advanced stages and high metastatic potential [24]. Despite advances in diagnosis and systemic treatment, the prognosis for patients diagnosed with GC, especially metastatic GC, remains poor [25]. To date, an optimal prognostic biomarker for GC has not been established. Herein, we confirmed the upregulation of *CRISPLD1* expression in GC samples and revealed its clinical significance, indicating its potential value in predicting GC prognosis.

CRISPLD1 is a member of the highly conserved CRISP protein family and has a molecular weight of approximately 56.9 kDa. It is expressed in lung fibroblasts and has been suggested as a novel biomarker for experimental pulmonary fibrosis. CRISPLD1 plays a role in facial morphogenesis, the folate pathway, and the response of chondrocytes to interleukin (IL)-1α-induced cellular stress [26,27]. According to GWAS studies, SNPs of CRISPLD1/CRISPLD2 are involved in the variation of folate pathway genes in non-syndromic cleft lip and palate [28]. Furthermore, in the treatment of coronary heart disease, the CRISPLD1 rs12115090 A > C polymorphism enhances the antiplatelet effectiveness of clopidogrel [29]. CRISPLD1 has been identified as a regulator of hematopoietic stem cell proliferation in mice. Moreover, it was observed to be regulated by mechanistic target of rapamycin kinase (mTOR) activation in the context of tuberous sclerosis complex-associated renal cell carcinoma gene alterations identified through whole-exome sequencing screening [13]. As a newly discovered molecule, its function in human tumors has not been reported. In this study, we found abnormal expression of *CRISPLD1* in various tumors based on the pan-cancer analysis using TIMER2.0. Additionally, analysis of the TCGA database revealed a significant correlation between abnormal *CRISPLD1* expression and clinical prognosis of GC. Furthermore, *CRISPLD1* expression levels showed significant correlations with T stage, overall survival events, age, and stage. Through *in vitro* experiments, it was observed that the downregulation of CRISPLD1 had a significant inhibitory effect on the proliferation and invasion of GC cells. Furthermore, in vivo studies showed that knockdown of CRISPLD1 suppressed the growth of GC tumors. These findings strongly suggest that CRISPLD1 acts as a tumor promoter in GC and could potentially be targeted for novel therapeutic interventions in the treatment of GC.

RETRACTED

To explore the potential mechanisms of CRISPLD1 in GC, we conducted differential gene expression analysis on GC samples from the TCGA and performed GO and KEGG functional enrichment analysis on the DEGs. The results revealed significant associations with the calcium and PI3K-AKT signaling pathways. Calcium ions are crucial signaling molecules in cells and have been shown to play a key role in regulating the malignant phenotype of tumor cells [30]. Calcium signaling is a critical regulatory factor for many cancer-related features, such as angiogenesis, invasiveness, and migration [31]. Therefore, we used flow cytometry analysis to demonstrate that *CRISPLD1* knockdown reduced the concentration of Ca^2+^ in GC cells. Additionally, fluorescence microscopy observation showed that *CRISPLD1* knockdown weakened the fluorescence intensity of the Ca^2+^ fluorescent probe in GC cells. Studies have shown that PTEN and cytosolic calcium homeostasis are two major upstream regulators of the AKT pathway, and their important roles in regulating AKT activity are well-documented [32]. We hypothesized that CRISPLD1 might inhibit the activation of the PI3K-AKT signaling pathway by regulating intracellular calcium levels. Western blotting analysis revealed that *CRISPLD1* knockdown significantly reduced the levels of p-PI3K and p-AKT in GC cells. It has been reported that some genes affect GC cell proliferation, invasion, and tumor angiogenesis through the PI3K/AKT/mTOR signaling pathway [33,34]. Given the strong evidence that CRISPLD1 positively regulates the levels of phosphorylated PI3K-AKT in GC, we speculated that CRISPLD1 promotes GC migration and invasion, at least in part, via the PI3K-AKT pathway. Consequently, treatment with a specific AKT activator (SC79) eliminated the inhibitory effect of *CRISPLD1* knockdown on GC cell migration and invasion, supporting the concept that CRISPLD1 mediates GC cell migration and invasion through the PI3K-AKT signaling pathway.

RETRACTED

## 5 Conclusion

Our study identified CRISPLD1 as a novel oncogenic molecule in GC, and its high expression is closely associated with tumor progression and clinical prognosis. Mechanistically, it might promote tumor cell progression by mediating intracellular calcium levels and activating the PI3K-AKT pathway, ultimately impacting the survival of patients GC. However, the direct mechanism of CRISPLD1's involvement in the Calcium signaling pathway is yet to be explored. This critical role of CRISPLD1 in tumor progression provides a theoretical basis to further understand the pathogenesis of GC and to develop novel therapeutic strategies.

## Funding statement

This work was supported by 10.13039/501100004731Zhejiang Provincial Nature Science Foundation of China (LR20H160001 to Wei Chen), Key R&D projects of Zhejiang Province (2021C03012 to Wei Chen), Young Qihuang Scholar of National Administration of Traditional Chinese Medicine (to Wei Chen), Zhejiang Provincial Traditional Chinese Medicine Science and Technology Project (2020ZZ004 to Wei Chen), 10.13039/501100001809Natural Science Foundation of China (81972693, 81802383, 81972674, 81673809 and 31900543)

## Data availability

The data that support the findings of this study are available on request from the corresponding author The data that support the findings of this study are available from the corresponding authors upon reasonable request.

## CRediT authorship contribution statement

**Liqiang Hu:** Data curation. **Jianghua Shi:** Writing – original draft. **Zichen Zhu:** Visualization. **Xuemei Lu:** Software. **Huibo Jiang:** Validation. **Hanyang Yu:** Writing – review & editing. **Hao Liu:** Project administration. **Wei Chen:** Writing – original draft, Conceptualization.

## Declaration of competing interest

The authors declare that they have no known competing financial interests or personal relationships that could have appeared to influence the work reported in this paper.

## Figures and Tables

**figs1:** 
